# A Joint Model for Macular Edema Analysis in Optical Coherence Tomography Images Based on Image Enhancement and Segmentation

**DOI:** 10.1155/2021/6679556

**Published:** 2021-02-17

**Authors:** Zhifu Tao, Wenping Zhang, Mudi Yao, Yuanfu Zhong, Yanan Sun, Xiu-Miao Li, Jin Yao, Qin Jiang, Peirong Lu, Zhenhua Wang

**Affiliations:** ^1^Department of Ophthalmology, The First Affiliated Hospital of Soochow University, Suzhou 215006, China; ^2^College of Information Science, Shanghai Ocean University, Shanghai 201306, China; ^3^The Affiliated Eye Hospital, Nanjing Medical University, Nanjing 210029, China; ^4^Eye Institute, Eye & ENT Hospital, Shanghai Medical College, Fudan University, Shanghai 200030, China

## Abstract

Optical coherence tomography (OCT) provides the visualization of macular edema which can assist ophthalmologists in the diagnosis of ocular diseases. Macular edema is a major cause of vision loss in patients with retinal vein occlusion (RVO). However, manual delineation of macular edema is a laborious and time-consuming task. This study proposes a joint model for automatic delineation of macular edema in OCT images. This model consists of two steps: image enhancement using a bioinspired algorithm and macular edema segmentation using a Gaussian-filtering regularized level set (SBGFRLS) algorithm. We then evaluated the delineation efficiency using the following parameters: accuracy, precision, sensitivity, specificity, Dice's similarity coefficient, IOU, and kappa coefficient. Compared with the traditional level set algorithms, including C-V and GAC, the proposed model had higher efficiency in macular edema delineation as shown by reduced processing time and iteration times. Moreover, the accuracy, precision, sensitivity, specificity, Dice's similarity coefficient, IOU, and kappa coefficient for macular edema delineation could reach 99.7%, 97.8%, 96.0%, 99.0%, 96.9%, 94.0%, and 96.8%, respectively. More importantly, the proposed model had comparable precision but shorter processing time compared with manual delineation. Collectively, this study provides a novel model for the delineation of macular edema in OCT images, which can assist the ophthalmologists for the screening and diagnosis of retinal diseases.

## 1. Introduction

Retinal vein occlusion (RVO) is one of the most common retinal vascular disorders, which is a significant cause of visual loss, affecting at least 16 million people globally [1, 2]. Macular edema is the major pathological feature of RVO caused by the accumulation of fluid in the macula due to impaired capillary perfusion and retinal ischemia. Serious macular edema can lead to vision loss in patients with RVO [3, 4]. Hence, early detection of macular edema can reduce the incidence of blindness in patients with RVO [5].

Optical coherence tomography (OCT) is a noninvasive technique, which has been used for clinical imaging and retinal visualization [6]. OCT images can provide important information on retinal internal structures and help in the detection of early symptoms of retinal pathology. It has been used for monitoring macular edema in many ocular diseases, such as age-related macular degeneration (AMD), diabetic macular edema (DME), and RVO [7–10]. The major benefit of OCT over other ocular testing techniques is that it can provide an objective and accurate visualization of early retinal syndromes [11]. However, OCT images often suffer from speckle noises. Speckle noises limit the contrast and the signal-to-noise ratio (SNR) of OCT images and cause difficulty in the segmentation of macular edema through direct observation or use of segmentation algorithms [12]. Moreover, manual segmentation of an edema region is often not objective and suffers from intersubject variations in the clinic. The screening of a huge amount of RVO patients is a tedious and time-consuming task [13]. Hence, developing a model to rapidly and accurately detect macular edema in OCT images is necessary.

Image enhancement is the first step in OCT image analysis. It can improve the visual appearance of an OCT image and provide a better transform representation for subsequent image processing. Currently, several algorithms have been successfully applied in many science, medical, and engineering fields [11–14]. Chong and Zhu used a block-matching 3D filter modified by the Morlet wavelet decomposition to sharpen OCT images [14]. Dong et al. developed a custom generative adversarial network (GAN) to denoise OCT images [15]. Sahu et al. applied an adaptive wavelet thresholding method for the enhancement and denoising of OCT images [16]. Hojjatoleslami and Avanaki proposed an OCT skin image enhancement through the attenuation compensation algorithm [17]. Other enhancement algorithms, including Lee et al.'s approach [18], regionally adaptive histogram equalization [19], median filtering, and homomorphic filtering [20] have also been used for OCT image processing. However, it is still a challenge to find the most suitable, accurate, faster, and robust algorithm for OCT image enhancement. Biological systems have the capability to adapt to changes by learning. Mimicking the system into algorithms introduces bioinspired algorithms, which can seek to solve computer science problems using the models of biology [21]. Retinal structures vary among individuals and among different disease conditions and stages. Thus, we used the bioinspired algorithm for OCT image enhancement due to its capability to adapt to changes by learning.

Image segmentation is the critical step for successful OCT image analysis. An active contour algorithm is a popular algorithm used for medical image segmentation [22]. The active contour algorithm can be categorized into two types including the edge-based algorithm and the region-based algorithm [23]. The geodesic active contour (GAC) algorithm is an edge-based algorithm [24]. The GAC algorithm delineates the target regions by utilizing edge stopping function (ESF) to stop the contour evolution on the boundaries [25]. However, this algorithm usually leads to a high level of noise, and the object is usually characterized by weak edges [26]. The Chan-Vese (C-V) active contour algorithm is a region-based algorithm [27, 28]. This algorithm has been used for the statistical intensity information to construct a stopping function [29]. Compared to an edge-based algorithm, the region-based model is less sensitive to the initialization of a contour and performs better in images with blurred edges [30]. However, the C-V algorithm is time-consuming because the average intensities inside and outside the contour should be computed at each iteration [31]. Many computer-aided systems have been proposed to assist ophthalmologists in clinical diagnosis in OCT images [32–38]. However, a computer-aided system depends on a mass of datasets and high-performance computing equipment, and it is not universal. The selective binary and Gaussian-filtering regularized level set (SBGFRLS) algorithm combines the merit of edge-based and region-based algorithms [22]. In the SBGFRLS algorithm, the signed pressure function (SPF) can efficiently stop the contours at the weak or blurred edges. Moreover, the exterior and interior boundaries can be detected no matter where the initial contour starts [39, 40]. However, the SBGFRLS algorithm is highly dependent on the quality of OCT images.

In this study, we proposed a joint model for the segmentation of macular edema in OCT images. The joint model adopts the bioinspired algorithm to enhance the quality of OCT images and uses the Gaussian-filtering regularized level set (SBGFRLS) algorithm to segment macular edema in OCT images. The SBGFRLS algorithm can efficiently stop the contours at weak or blurred edges. The exterior and interior boundaries can be detected no matter where the initial contour starts. Moreover, this joint model is very simple to use because it is not highly dependent on multiple training OCT images and complex computational devices.

## 2. Materials and Methods

### 2.1. Materials

This study followed the tenets of the Declaration of Helsinki and approval was obtained by the Institutional Review Ethics Committee of the Affiliated Eye Hospital, Nanjing Medical University. The patients with RVO who presented to the hospital between May 1, 2018 and June 30, 2019 were included. All subjects gave their informed consent before inclusion. All patients were required to undergo OCT scanning with spectral domain OCT (RTVue, Optovue Inc., USA). Visual interpretation of edema was performed by retinal specialists. These OCT images were centered on the macula with an axial resolution of 10 *μ*m and a 24-bit depth and were acquired in 2 seconds, covering a 4 × 4 mm area. Raw OCT images were exported from the imaging system for subsequent analysis, including image quality enhancement using the bioinspired algorithms and edema segmentation by SBGFRLS.

### 2.2. Methodology

The joint model for the segmentation of macular edema consists of two main steps: (1) image enhancement using bioinspired algorithms (including speckle noise reduction by Gaussian filter (GF) and structure-preserving guided retinal image filtering (SGRIF)) and contrast enhancement using the Retinex algorithm, and (2) segmentation of macular edema by SBGFRLS.  Figure 1 is the flowchart of the joint model for the delineation of macular edema (Figure 1).

#### 2.2.1. Step 1: OCT Image Enhancement Using the Bioinspired Algorithm

Taking the original OCT images as the input data, the quality of OCT images was enhanced using the bioinspired algorithm, including speckle noise reduction and contrast enhancement. Firstly, the speckle noises in OCT images were reduced by GF and SGRIF algorithms. Here, the original OCT image (*I*(*x*, *y*)) was expressed as follows:

(1) $$\begin{array}{c} I\left(x,y\right)=S\left(x,y\right)*N_{s}\left(x,y\right)+N_{b}\left(x,y\right), \end{array}$$

where *S*(*x*, *y*) donates the desired noise-free image information, *N*_*s*_(*x*, *y*) and *N*_*b*_(*x*, *y*) donates the speckle and background noises, respectively. Equation (1) was rewritten in logarithmic compression:

(2) $$\begin{array}{c} \text{Log}I\left(x,y\right)=\log S\left(x,y\right)+\log N\left(x,y\right), \end{array}$$

where *N*(*x*, *y*) is approximated to the additive white noise. In equation (2), the speckle noise was changed from multiplicative to additive.

According to GF, the speckle noises were divided into a real part and an imaginary part independently and identically [41]. The two-dimensional digital Gaussian filter is denoted as follows:

(3) $$\begin{array}{c} G\left(x,y\right)=\frac{1}{\sqrt{2\pi \sigma }}\exp\left(-\frac{x^{2}+y^{2}}{2\sigma^{2}}\right), \end{array}$$

where *σ*^2^ is the variance of GF. Here, a 5 × 5 filter kernel size was adopted in the following experiments. According to GF, the OCT images were smoothed and denoised. Then, the edge of OCT images were preserved by SGRIF [42].

Equation (4) shows the objective function of a global structure transfer filter:

(4) $$\begin{array}{c} \left(\lambda A+D_{x}^{T}D_{x}+D_{y}^{T}D_{y}\right)O=\lambda I+D_{x}^{T}V^{h}+D_{y}^{T}V^{v}, \end{array}$$

where *A* is the identity matrix; *O* indicates the output image; *I* indicates the input image; *λ* is the parameter controlling the trade-off between the two terms; *D*_*x*_ and *D*_*y*_ are discrete differentiation operators; *V* = (*V*^*h*^, *V*^*v*^) is a guidance vector field of the OCT image. Output OCT images were enhanced by the next contrast enhancement step.

According to the Retinex algorithm, the image was taken as a multiplication of illumination and reflectance of the object. The illumination characteristics of images depended on the source of illumination. The reflectance characteristics of images depended on the nature of the object [43, 44]. The image is expressed as follows:

(5) $$\begin{array}{c} I\left(x,y\right)=R\left(x,y\right)\cdot L\left(x,y\right), \end{array}$$

where the range of *I*(*x*, *y*) is between 0 and 255. *R*(*x*, *y*) denotes the reflectance of the image, and the range is between 0 and 1. *L*(*x*, *y*) denotes the illumination characteristics of the image, and the range is between 0 and 255.

Here, a single-scale Retinex (SSR) was adopted to enhance the contrast of the OCT image calculated by the following parameters:

(6) $$\begin{array}{c} R_{i}\left(x,y\right)=\ln I_{i}\left(x,y\right)-\ln\left[G\left(x,y\right)*I_{i}\left(x,y\right)\right], \end{array}$$

where *I*_*i*_ represents the *i*th color channel of an image, and the convolution operator is denoted by ∗. *R*(*x*, *y*) represents the output of the respective Retinex. *G*(*x*, *y*) denotes the surround function represented as follows:

(7) $$\begin{array}{c} G\left(x,y,c\right)=K\cdot \exp\left(-\frac{x^{2}+y^{2}}{c^{2}}\right), \end{array}$$

where *c* represents the scalar value and could be called either the surround space or the Gaussian space constant. The selection of *K* is based on

(8) $$\begin{array}{c} \int \int G\left(x,y,c\right)dxdy=1. \end{array}$$

The output images were used as the input image for subsequent segmentation.

#### 2.2.2. Step 2: Edema Segmentation by SBGFRLS Algorithm

The SBGFRLS algorithm was calculated by the level set formulation and SPF function. Its level set formulation is described as follows:

(9) $$\begin{array}{c} \frac{\partial \phi }{\partial \phi }=\text{SPF}\left(I\cdot \alpha \left|\nabla \phi \right|\right), \end{array}$$

where *ϕ* is the level set and *t* is time. *I* is the input image. *α* is the balloon force parameter. ∇*ϕ* is the gradient operator of *ϕ*. The range is [−1, 1]. This function modulates the signs of pressure forces inside and outside of the regions of interest, so that the contour shrinks when outside the object, or expands when inside the object. The SPF function of the SBGFRLS algorithm is shown as follows:

(10) $$\begin{array}{c} \text{SPF}\left(I\right)=\frac{I-\left(c_{1}+c_{2}/2\right)}{\max\left(\left|I-\left(c_{1}+c_{2}/2\right)\right|\right)}, \end{array}$$

where *c*_1_ and *c*_2_ are computed by equation (11). *c*_1_ and *c*_2_ are the mean gray values of the inside and outside curves.

(11) $$\begin{array}{c} \left\{\begin{array}{c} c_{1}\left(\phi \right)=\frac{\int_{\Omega }I\left(x,y\right)\cdot H\left(\phi \right)dxdy}{\int_{\Omega }H\left(\phi \right)dxdy},\\ c_{2}\left(\phi \right)=\frac{\int_{\Omega }I\left(x,y\right)\cdot \left(1-H\left(\phi \right)\right)dxdy}{\int_{\Omega }\left(1-H\left(\phi \right)\right)dxdy}, \end{array}\right. \end{array}$$

### 2.3. Implementation of Pseudocode

The implementation of pseudocode for the proposedmodel was shown in Algorithm 1.

## 3. Results

We conducted three different experiments to evaluate the performance of the joint model. First, we evaluated the enhancement performance of the joint model. Then, we compared the segmentation performance of the joint model against conventional level set algorithms, including GAC and C-V. Finally, we compared the segmentation performance of the joint model against manual interpretation.

### 3.1. Evaluation of Enhancement Performance of the Joint Model

12 original images and their enhancement images were compared to evaluate the enhancement performance. As shown in Figure 2, the enhancement processing removed a fair amount of speckle noises and preserved the fine edges and detailed structures. The edema region and background region had a higher contrast in the enhanced images.

Taking the contrast-to-noise ratio (CNR) and equivalent number of looks (ENL) as the evaluation index of image quality [14], the quality differences between original images and enhanced images were estimated. CNR and ENL were defined by

(12) $$\begin{array}{c} \text{CNR}=\frac{1}{R}\left(\overset{R}{\underset{r=1}{\sum }}\frac{\left(\mu_{r}-\mu_{b}\right)}{\sqrt{\sigma_{r}^{2}+\sigma_{b}^{2}}}\right),\\ \text{ENL}=\frac{1}{R}\left(\overset{H}{\underset{h=1}{\sum }}\frac{\mu_{h}^{2}}{\sigma_{h}^{2}}\right), \end{array}$$

where *μ*_*b*_ and *σ*_*b*_^2^ represents the mean and the variance of background noise, respectively. *μ*_*h*_ and *σ*_*h*_^2^ represents the mean and the variance of the homogenous region of interest, respectively.

Figure 3 showed the comparison evaluation metrics of image quality, CNR and ENL, respectively. The joint model had greater metrics of CNR and ENL. The joint model generated better visual effects of edge preservation and speckle noise reduction in enhanced OCT images compared with original images.

The comparison results of macular edema segmentation using the SBGFRLS algorithm between the original OCT image and the enhanced OCT image are shown in Figure 4. In Figure 4(a), the false positives were detected near areas containing low contrast. Since the gray value was similar to the edema region, the algorithm perceived these areas as “abnormal,” thus resulting in false positive classifications.  Figure 4(b) shows the smooth boundary of the retina and the accurate segmentation result of macular edema in an enhanced OCT image.

### 3.2. Comparison Result of Edema Segmentation between the Joint Model and Conventional Level Set Algorithms

We compared the segmentation performance and efficiency of the joint model against the conventional level set algorithms, including GAC and C-V (Figure 5). The GAC algorithm could not delineate the regions of the retina and edema (Figure 5(a)). The C-V algorithm obtained both the retina region and the edema region. However, the accuracy rate of segmentation was very low (Figure 5(b)). By contrast, the joint model obtained an accurate segmentation result of the retina region and the edema region (Figure 5(c)).

We calculated the processing time and the number of iteration times to evaluate the efficiency of edema segmentation. As shown in Table 1, compared with C-V or GAC algorithm, the joint model greatly reduced the processing time and the number of iteration times. The processing time in the joint model was about 6556 times or 15556 times less than the time in the GAC or C-V algorithm. Compared with the C-V or GAC algorithm, the number of iterations of the joint model was reduced by 181 times and 51 times, suggesting that the joint model is more efficient in segmentation than other level set algorithms.

### 3.3. Comparison of Segmentation Performance of Macular Edema between the Joint Model and Manual Interpretation

We then selected 1000 OCT images and compared the segmentation performance of the edema region between the joint model and manual interpretation. At first, these OCT images were carefully judged by three retinal experts with more than 10-year clinical experience. The consistent segmentation results were used as the gold standard. We then compared the segmentation performance between the joint model and manual interpretation by an additional 5 clinicians using the following indicators: accuracy, precision, sensitivity, specificity, Dice's similarity coefficient, IOU, and kappa coefficient [45]. It is generally accepted that if Dice's similarity coefficient reaches higher than 0.70, then it indicates excellent agreement. Dice's similarity coefficient could reach 0.97 in the joint model, suggesting that the joint model can achieve similar segmentation performance as manual interpretation. Moreover, the joint model had higher accuracy (99.7%), precision (97.8%), sensitivity (96.0%), specificity (99.0%), IOU (94.0%), and kappa coefficient (96.8%). Compared with manual interpretation, the joint model has a comparable performance for macular edema segmentation (Table 2). Furthermore, the joint model spent less CPU time which was about 55 times less than the time of manual segmentation.  Figure 6 shows the representative segmentation results of the RVO region between the joint model and manual interpretation.

## 4. Discussion

RVO is one of the most common retinal disorders [46]. Macular edema is the major cause of vision loss in patients with RVO [47]. Early detection of macular edema can reduce the incidence of blindness. In this study, we proposed a joint model which could detect macular edema in OCT images. The image-enhanced algorithm was used to improve the contrast of OCT images and maintain the edges of macular edema. Then, the SBGFRLS algorithm was used to delineate edema regions in the OCT images.

Since OCT images take advantage of low-coherence interferometry, the occurrence of noises in OCT images are inevitable [48, 49]. The noises of OCT images can destroy the quality of images and affect the results of segmentation [50]. The major goal of noise reduction is to remove image noises without losing the critical details in OCT images [51, 52]. OCT denoising has been achieved by Bayesian least-squares estimation [53] and spatially adaptive wavelet filter [54]. However, these methods cannot effectively maintain the fine edges like edema regions in the retinal structure. In this study, GF and SGRIF algorithm was used for OCT image denoising and structure preservation. The Retinex algorithm was used for OCT image enhancement. The enhanced OCT image showed significant improvement in both CNR (more than 0.95 dB on average) and ENL (more than 12 times).

We then used the SBGFRLS algorithm for edema segmentation. Compared with the GAC and C-V methods, the SBGFRLS algorithm had higher efficiency in edema segmentation as shown by decreased mean processing time (s) and mean iteration times (time). Accuracy, precision, sensitivity, specificity, Dice's similarity coefficient, IOU, and kappa coefficient were calculated to evaluate the performance of edema segmentation. Dice's similarity coefficient is a dimensionless ratio where 1 corresponds to the perfect match between the images being compared. Dice's similarity coefficient higher than 0.70 indicates excellent agreement [45]. The Dice's similarity coefficient of the proposed model can reach 0.97. The accuracy, precision, sensitivity, specificity, IOU, and kappa coefficient can reach 99.7%, 97.8%, 96.0%, 99.0%, 94.0%, and 96.8%, respectively, suggesting that the proposed model has a similar performance of edema segmentation as ophthalmologists.

Although the proposed joint model can efficiently segment the regions of macular edema in OCT images compared with state-of-the-art methods, there are still some constraints and limitations in the practical applications. This model can only segment the outline of macular edema but it cannot calculate the depth and volume of the macular edema region, which are also important information for disease diagnosis. Given great variations in disease pathology, the quality of OCT images is also highly varied. Deep learning can help to identify, classify, and quantify the pathological features in OCT images to increase the accuracy and efficiency of segmentation. Our proposed model did not consider the application of deep learning. In the future, we will augment the dataset of OCT images, enhance computer configuration, develop new deep learning algorithms, and design a system to improve the accuracy and efficiency of edema segmentation in OCT images.

## 5. Conclusions

This study developed a joint model for the analysis of macular edema in OCT images based on image enhancement and segmentation. An image enhancement algorithm improves the contrast of images and maintains the edges of edema regions. The SBGFRLS level set algorithm can efficiently delineate edema regions in OCT images. This joint model will assist ophthalmologists in the segmentation of the edema region and enhance the efficiency of RVO diagnosis.

## Figures and Tables

**Figure 1:** Flowchart of joint model for macular edema delineation.

**Figure 2:** OCT image enhancement processing. (a) Original OCT image; (b) Smoothed OCT image by GF; (c) Denoised OCT image by SGRIF; (d) Enhanced OCT image.

**Figure 3:** Comparison of evaluation metrics of image quality.

**Figure 4:** Segmentation performance comparison of macular edema using the SBGFRLS algorithm between original images and enhanced images: (a) segmentation result of macular edema in the original OCT image; (b) segmentation result of macular edema region in the enhanced OCT image. Red curves indicate the retinal region, and green curves indicate the edema region.

**Figure 5:** Comparison of segmentation performance of macular edema between the proposed model and two conventional level set algorithms: (a) GAC algorithm; (b) C-V algorithm; (c) the joint model. The images show the result of edema segmentation. Red lines are used to label the retinal region (ROI). Green lines are used to label the edema region.

**Figure 6:** Comparison of segmentation performance of macular edema between the joint model and manual interpretation. (a–e) Original OCT images with RVO pathology. (f–j) Segmentation results of macular edema by the joint model. (k–o) Segmentation results of macular edema by five different clinicians. Red lines are used to label the retinal region (ROI). Green lines are used to label the macular edema.

**Algorithm 1:** A joint model for macular edema segmentation in OCT images.

**Table 1:** Mean processing time and iteration times for the segmentation of macular edema by GAC, C-V, and the joint model.

Mean	GAC	C-V	The joint model
Processing time (s)	34690 ± 3933^∗^	82298 ± 7794^∗^	5.3 ± 0.6^∗^
Iteration times (time)	8560 ± 477.4^∗^	2480 ± 148.3^∗^	47 ± 4.7^∗^

All data were shown as mean ± SD. *n* = 20. The significant difference was calculated by one-way ANOVA. ^∗^*P* < 0.05 versus the joint model.

**Table 2:** Comparison of segmentation performance of macular edema between the joint model and five different clinicians.

	Accuracy	Precision	Sensitivity	Specificity	Dice	IOU	Kappa	Processing time (s)
Clinician 1	95%	97%	95%	97%	97%	93%	94%	1500
Clinician 2	96%	98%	98%	96%	96%	95%	96%	1200
Clinician 3	96%	97%	89%	94%	87%	92%	95%	2020
Clinician 4	97%	95%	91%	95%	93%	89%	94%	1760
Clinician 5	95%	98%	93%	95%	92%	84%	91%	1880
Joint model	99.7%	97.8%	96.0%	99.0%	96.9%	94.0%	96.8%	30

## Data Availability

The data used to support the findings of this study are included within the article.
